# Real-Time Heart Arrhythmia Detection Using Apache Spark Structured Streaming

**DOI:** 10.1155/2021/6624829

**Published:** 2021-04-22

**Authors:** Sadegh Ilbeigipour, Amir Albadvi, Elham Akhondzadeh Noughabi

**Affiliations:** Department of Information Technology Engineering, Industrial and Systems Engineering Faculty, Tarbiat Modares University, Tehran, Iran

## Abstract

One of the major causes of death in the world is cardiac arrhythmias. In the field of healthcare, physicians use the patient's electrocardiogram (ECG) records to detect arrhythmias, which indicate the electrical activity of the patient's heart. The problem is that the symptoms do not always appear and the physician may be mistaken in the diagnosis. Therefore, patients need continuous monitoring through real-time ECG analysis to detect arrhythmias in a timely manner and prevent an eventual incident that threatens the patient's life. In this research, we used the Structured Streaming module built top on the open-source Apache Spark platform for the first time to implement a machine learning pipeline for real-time cardiac arrhythmias detection and evaluate the impact of using this new module on classification performance metrics and the rate of delay in arrhythmia detection. The ECG data collected from the MIT/BIH database for the detection of three class labels: normal beats, RBBB, and atrial fibrillation arrhythmias. We also developed three decision trees, random forest, and logistic regression multiclass classifiers for data classification where the random forest classifier showed better performance in classification than the other two classifiers. The results show previous results in performance metrics of the classification model and a significant decrease in pipeline runtime by using more class labels compared to previous studies.

## 1. Introduction

### 1.1. Healthcare Context

Modern healthcare has become a process that can provide data analysis with the support of various sources. For example, patients who need remote monitoring or home monitoring and wireless and wearable remote sensors can generate the data needed to manage the health of these patients. Also, big data can lead to more accurate decisions and changes in the providing of health care services [1]. With the increase in healthcare data, new technologies have been developed to process them [2]. Discovering knowledge and accessing useful medical information that can improve services, reduce patient and hospital costs, and save patient lives is possible through the analysis of these data [3, 4]. In the field of cardiovascular disease, the use of big data analysis is increasingly used in health care than in the past. Intelligent sensors and smartphones are designed to receive physiological information and the patient's ECG signal, providing real-time detection of deadly cardiac arrhythmias and early warning [1]. ECG data, which are the most important medical health data, have features such as high speed and sequential production. With these features, a big data platform can be used to real-time analyze and detect cardiac arrhythmias [5]. The most important cardiac arrhythmias that can be diagnosed through ECG are atrial fibrillation (AF) and right bundle branch block (RBBB) arrhythmias [6, 7]. AF is one of the most prevalent cardiac arrhythmias [6]. In addition to heart failure, it can lead to stroke in patients; it has a profound effect on patients' lives and is a threat to their lives [8, 9]. But the right block of the heart electrical conduction system responsible for activating the right ventricle is called the right bundle branch block.

During RBBB arrhythmia, impulses passed by the right bundle branch are unable to activate the right ventricular. Many techniques have been used in batch mode and static environment for AF detection [10, 11]. However, there are generally many methods of stream processing in real-time mode. These are database, mining, or tool-based methods. Sampling, sketching [12], and approximation [13] are the types of database-based techniques. Mining methods refer to machine learning algorithms that are essentially designed for stream mining [14, 15]. Finally, the tool-based methods allow working with the data stream. Massive Online Analysis (MOA) [16] and Rapid Miner [17] Streaming Computation Engines [18] like Apache Spark Streaming, Apache Spark Structured Streaming, apache storm, etc. are tool-based methods for stream processing. Streaming Computation Engines, unlike traditional tools, are capable of supporting parallel and distributed computing.

Several methods have been developed for the real-time diagnosis of AF and RBBB arrhythmias. The Pan-Tampkins [19] algorithm is a mining-based technique for real-time QRS-complex detection of ECG signal that can be used for real-time detection of AF [20] and RBBB [21] beats. Some tool-based methods have been proposed and have used a big data platform for real-time AF [22] and CHF detection [5].

In this paper, we have implemented a novel machine learning pipeline using the Apache Spark Structured Streaming Processing Engine for real-time detection of AF and RBBB arrhythmias in the ECG signal. This approach is a tool-based approach that has not yet been implemented with a Spark Structured Streaming able to support distributed and parallel computing. We also were able to make a real-time diagnosis of more class labels of cardiac arrhythmias with less time and high performance through the use of weaker hardware resources compared to previous studies.

The Apache Spark Structured Streaming is a new stream processing engine built on the open-source Apache Spark platform that enables real-time data processing. Besides, the Structured Streaming Processing Engine is based on Data Frame/Dataset API built on the Spark SQL Library and can address other big data platform constraints [23]. Therefore, it is possible to use SQL commands on streaming data. Our study is the first approach that uses this processing engine for real-time cardiac arrhythmias detection. With theories defined in this processing engine, the Spark Structured Streaming compared to other stream processing tools provides new capabilities with data frame API that make it reliable on real streaming [24]. The following are the features:

1. I/O optimization: unlike other big data tools in stream processing and existing algorithms, Structured Streaming can receive data from multiple inputs and send the result to different output sinks. Depending on the need of the application, these capabilities can significantly reduce the delay in sending results to the user
2. Performance, throughput, and latency: studies show that Structured Streaming has higher performance than other streaming systems. Recent research [24] has compared Structured Streaming with other streaming platforms developed in a similar infrastructure. The results show that Structured Streaming is more efficient than other systems in terms of performance and throughput and latency [24]. For example, Structured Streaming has a maximum throughput of 65 million records per second, which is twice as much as Kafka Stream and Apache Flink. This high performance in Structured Streaming is only due to the storage of streaming data in a compressed format by the Spark SQL engine [24]. Therefore, SQL commands can significantly reduce the final workload of the system [25]. On the other hand, by providing different types of output generation modes (Append, Update,…), it produces much less delay in producing results in processing similar data than other stream processing tools [23]
3. User-friendly: Structured Streaming facilitates the implementation of incremental queries for different applications by providing a set of concepts such as event-time, watermark, processing time, and trigger [24]. Although other streaming systems such as Apache Spark Streaming, Google Data Flow [26], and Apache Flink [27] offer various functional functions, they require the user to define a physical layout of the consecutive tasks. On the other hand, Structured Streaming users define their stream-processing logic using the powerful UDF State full operators [24]
4. Powerful functions: Structured Streaming provided a set of powerful functions by data frame API that enables users to implement different policies for joining stream, batch, or interactive processes together in the same code. These functions have not yet been developed on other platforms [24]. Although the Apache Flink platform recently supports table API, it still lacks many of the Structured Streaming features for real-time data stream analysis [24]
5. Guaranteed exactly-once delivery: Structured Streaming guarantees that if any defect occurs in the streaming system, it will deliver the results exactly once [24]
6. Fault tolerance: our streaming system is fault-tolerant with the concept of exactly-once delivery and ensures that data is not lost if the system crashes. Hence, by rebooting the system, results are generated immediately after the failure point [24]

### 1.2. Related Works

As mentioned in the previous section, many approaches have been proposed to diagnose cardiac arrhythmias in the literature. In [28], AF can be detected using a smartphone, and the proposed algorithm measures the RR interval by calculating the QRS complex and uses it to classify the ECG signal beats. In this study, the results of accuracy, specificity, and sensitivity of AF detection were 97%, 100%, and 93%, respectively. Researchers in [6] have used several statistical methods to separate AF beats from normal beats in a mobile phone. The authors have claimed that their approach is real-time realizable and the accuracy of the results by combining all statistical methods was 99%.

Many approaches based on RR interval in heartbeats have been proposed for AF detection; for example, researchers in [29] calculated the RR interval and difference between these RR intervals and comparison difference between coefficients of deviation with their standard deviation coefficients, have detected AF in real time, and have achieved the best results for the sensitivity of 94.4% and specificity of 97.2%.

Besides, the RR interval and Markov model is another method used to obtain RR Markov score for heartbeat classification and real-time detection of AF arrhythmia [30]. Researchers have used MIT/BIH database to validate the proposed algorithm and have achieved 92% sensitivity and 97% positive predictive value. Another algorithm for the real-time detection of AF arrhythmia based on its general specifications has been developed which uses three statistical techniques, namely, RMSSD, TPR, and Shannon Entropy, to identify these characteristics. They have used two different databases to validate the results and have achieved a sensitivity of 90.2% and specificity of 91.2% in AF arrhythmia detection combination with other arrhythmias [31].

Another approach proposed for the real-time detection of cardiac arrhythmias is to train a heartbeat classification model in an offline fashion to each specific patient and then apply it in an online mode to real-time patient monitoring [32]. An approach based on active learning to construct a patient-specific detector and real-time AF detection is presented in [33]. In this research, by extracting R-peak, computed consecutive RR intervals are used to construct feature vectors and training classifiers (SVM). After testing the three different classifiers, the best mean performance was obtained for all patients, including 91.96%,84.63%, and 94.38% for accuracy, sensitivity, and specificity, respectively. Heartbeat classification and automatic arrhythmia detection including AF and RBBB using two supervised and unsupervised machine learning techniques are presented in [34]. In this approach, after extracting several morphological features from each heartbeat, they are clustered to reduce the probable error and then labeled using the rule-based classification technique. Based on the results of this study, for AAMI-defined classes, the sensitivity and positive predictive value for the supraventricular class were 94.63% and 96.79%, respectively, and those for the ventricular class were 87.17% and 83.98%, respectively.

In recent years, several offline and online methods for diagnosing cardiac arrhythmias have been proposed in the literature. In a recent study proposed by Ghosh et al. [35] for offline cardiac arrhythmias detection, the extraction of ECG signal coefficients was used to evaluate the fractional norm(FN) properties in different subbands of a multirate cosine filter bank architecture. The obtained FNs were used to teach a deep learning model for detecting AF arrhythmia. In this study, the classification metrics were obtained for only two class labels with accuracy, sensitivity, and specifications of 99.4, 98.77, and 100%, respectively.

Deep learning models have been widely used to diagnose cardiac arrhythmias so far. These models have been able to partially compensate for the shortcomings of traditional methods in signal feature extraction. In the approach proposed in [36], the development of a multiscale convolutional neural network architecture is used to classify cardiac arrhythmias through multidimensional learning of ECG signal properties. This method is a multiclass classification method. Unlike previous methods, it can extract more important features from the signal. This feature makes it possible to differentiate between arrhythmia classes so that the model can more easily distinguish different beats from each other. Researchers evaluate the designed model with two different data sets and calculate the best F-score value equal to 84.1%. The authors claim that this value is higher than the previous state-of-the-art methods. A real-time cardiac arrhythmias detection approach based on nonlinear morphological features is proposed to detect rare morphological features in [37]. In this research, the MIT/BIH database and AAMI recommendation have been used to evaluate the proposed algorithm. Also, the beats are classified using an ensemble majority-vote-based approach. The classification metrics are calculated separately for each arrhythmia class. In this study, the average sensitivity and False Positive Rate measures for the three types of arrhythmias were 74.2% and 11.6%, respectively.

Mahmud et al. proposed an offline method for automatic cardiac arrhythmias detection based on AAMI annotation [38]. This approach uses a traditional methodology for ECG R-peak detection and then used a data augmentation technique to fix the class imbalance problem. In this study, researchers first design a structural unit based on pointwise temporal convolution and then develop a new depthwise temporal convolution architecture based on the convolutional neural network to improve unit performance. In this approach, the designed deep learning architecture can predict arrhythmia classes with 99% classification metrics.

Researchers in [39] implemented a solution to deal with S-type arrhythmias ectopic in AAMI annotation by two steps. In the first step, all fusion, ventricular, and unknown arrhythmias are detected using a deep dual-channel convolutional neural network. In the second step, a central-toward LSTM supportive model (CLSM) is designed to distinguish S-type arrhythmias from normal beats. The inputs of the CLSM model are the temporal features of the beats. Besides, researchers use a rule-based data augmentation method to solve the class imbalance problem and lack of input data for training the deep learning model. The overall accuracy of the system is 97.7%, and the recall and precision measures for detecting S-type beats are 85.6 and 65.7%, and those for the normal class are 98.2 and 99.4%, respectively.

## 2. Materials and Methods

### 2.1. Experiment Data

In this study, we develop a stream processing pipeline for the real-time detection of atrial and RBBB arrhythmias using segmentation and online features extraction of ECG signal and online classification using a random forest machine-learning algorithm.

A useful tool that physicians can use daily to examine patients is the electrocardiogram (ECG). These signals are often used to diagnose heart abnormalities and arrhythmias and to measure the electrical activity of the heart over a while. The ECG data required for the research is data collected from the well-known database MIT/BIH. The sampling frequency of the recorded signal from all patients is 360 Hz, and we have implemented our computation based on this sampling rate. The signal is recorded from two channels, where, according to the anatomical features of the patient in most of the recordings, two LEDs II and V1 have been used. In this database, most of the *R* peaks in the beats are marked and the type of beats is interpreted and recognized, which can be used in the training stage to train the machine learning model.

As mentioned in the previous section, this study considers three labels of beats for diagnosis based on MIT/BIH database labeling, including normal beat and also atrial and RBBB arrhythmia beat. But according to the AAMI recommendation for MIT/BIH database, all beats are placed in five superclasses, the RBBB beats are in the normal superclass, and the atrial arrhythmia is in the supraventricular superclass.  Table 1 shows the number of samples considered for each label along with the corresponding record from the database. The number of samples in Table 1 is calculated based on the 360 Hz sampling rate of the signal in the MIT/BIH database. Besides, a separate record for sampling is provided for each class label in this study. For example, the 205 and 115 records for the normal class label, the 118 and 124 records for the RBBB arrhythmia class label, and the 232 records for the atrial arrhythmia class label are based on the MIT/BIH database record annotations.

### 2.2. Data Preprocessing

Before processing data to analyze and arrhythmias detection, the data must be preprocessed to obtain reliable information. Data preprocessing consists of several steps that are performed to prepare the data for final processing and classification. In a real-time analysis, all the preprocessing steps are implemented online and the output of each stage provides input for the next step. In this study, we have implemented an online pipeline for running data preprocessing stages of ECG data on the Apache Spark platform. To do this, we used the Pandas-UDF technique in Spark, using which the traditional data mining functions and instructions can be run on the Apache Spark platform. Finally, the pipeline is built, using a spark structured stream processing engine that runs on ECG test data.

The data preprocessing step involves the steps of removing noise from the signal, R-peak detection, segmentation, and finally feature extraction. After performing the data preprocessing steps, the extracted features are classified in the final processing step for arrhythmia detection.  Figure 1 shows the block diagram of the data preprocessing steps and classification where the raw ECG data is segmented after the denoising and the R-peak detection as the unit beat, and in the last step by extracting the basic feature of each segment, the number of samples per segment is reduced to 25 samples. Finally, the extracted feature is classified by the classifier for arrhythmia detection in the final processing step.

### 2.3. ECG Denoising

The first step in data processing is to remove noise and artifacts from the data. Medical data, such as the ECG signal, may be exposed to a variety of noises depending on environmental conditions, which can affect the accuracy of this data. Therefore, before extracting the features of the ECG signal, we must remove this noise to obtain reliable signal data without distorting or missing the original information. We used the band-pass filter method, the Finite Impulse Response (FIR) to filter and eliminate noise from the ECG signal. The FIR band-pass filter is widely used for many digital signal processing applications. This filter has two features of the linear phase and high stability. The linear phase feature is used to design each amplitude-frequency characteristic, which is vital for the real-time processing of the digital signal.

### 2.4. R-Peak Detection

Each heartbeat is made up of several waves that are generated by electrical stimulation in the heart, and inside one beat, it represents the time evolution of an electrical cycle of the heart. Each arrhythmia causes a change in one or more of these waves. By identifying and measuring these changes, different arrhythmias can be detected. The most important part of a heartbeat is the QRS complex, which involves the waves of the *Q*, *R*, and *S*, and as a single event, they form the largest wave of a normal heartbeat.

At this stage of our research, since each heartbeat contains one QRS complex, we online detected the *R* points that make up the highest points in the QRS complex to find the single heartbeat. Using these points, we will be able to convert a large file of the ECG signal into unit beats in the next step with the segmentation technique. It is very important to accurately identify the *R* points of the ECG signal because it allows us to detect the beats, and this greatly affects the final results of the diagnosis of cardiac arrhythmias.  Figure 2 shows the results of the first and second stages of data preprocessing, in which a portion of the raw signal of the ECG is filtered to remove noise and the *R* peaks are detected.

### 2.5. Segmentation

As mentioned earlier, the purpose of segmentation operations is to break a large record from the ECG data to achieve single heartbeats with a fixed number of samples. In this preprocessing stage of the data, we convert the filtered ECG signal of the previous step into beats using the R peaks detected through the segmentation technique. In various studies, the number of samples of a heartbeat with a sampling rate of 360 Hz is randomly considered from 144 to 432 samples. In this study, we considered 200 samples for each beat, one sample for R-peak, 69 samples before R-peak, and 130 samples after R-peak, forming samples for each beat. The accuracy of segmentation is also important because if the number of samples is not considered appropriate for a single beat, important beat information may be lost, and then the accuracy of the final results of the arrhythmia detection will be reduced.

Figure 3 shows a normal beat after segmentation, with a sample number of 200, and the main information and basic features of the signal are preserved.

### 2.6. Feature Extraction

A cardiac signal cycle is composed of T-QRS-P waves. Useful clinical information is specified in an ECG signal at distances and amplitudes defined by its waves [40]. This information is divided into two categories: morphological and temporal features [40]. Morphological features are important morphological parameters including the QRS-complex duration, the PR wave distance, and the *T* segment. On the other hand, the temporal properties constitute a vector of signal statistical characteristics.

The purpose of feature extraction is to find as few features as possible in the ECG signal, which enables successful and efficient detection of the anomaly. Therefore, using an accurate and fast method for automatic feature extraction of ECG signals is of particular importance. What plays a key role in correctly diagnosing cardiac arrhythmias is the feature extracted from the ECG signal. The purpose of feature extraction is to find as few features as possible in the ECG signal to provide a successful and efficient diagnosis of arrhythmia.

In this research, we have used the discrete wavelet transform algorithm [41] up to 4 levels of decompositions to extract the signal statistical characteristics. This significantly reduces the number of original heartbeat samples while retaining useful information. Therefore, this action will reduce the delay in the classification process in the next step. In the discrete wavelet transform algorithm to discrete a signal with high sampling frequency to lower levels, the main signal first passes through a high-pass filter and then through a low-pass filter. After filtering, half of the signal samples are removed based on the Nyquist theorem [41]. This action indicates a level of decomposition. The above process, also known as subband encoding, is repeated for further decomposing the signal at higher levels. The samples and the frequency band are halved at each decomposition level [41]. The input of the current step is the previous output of the low-pass filter [41]. In this study, we reduced the number of 5-second epoch samples after segmentation from 200 samples to 25 main samples per beat with four levels of decomposition. In the classification stage, the decomposed epochs are sent to train the classification models.

The initial and reliable method used in the literature to extract the feature and useful information from statistical characteristics of the ECG signal is to reduce the signal samples by sampling the signal in the time domain and receiving the (*n*) sample *a*(*t*_1_), *a*(*t*_2_), ..., *a*(*t*_n_) and construct a vector(*A*) (equation (1)) from them [42].

(1) $$\begin{array}{c} A=\left[a1,a2,\ldots ,an\right]=\left[A\left(t1\right),A\left(t2\right),\ldots ,A\left(tn\right)\right], \end{array}$$

where *a*(*ti*) is a random variable vector.

To access signal information and build a vector *A*, the signal can be decomposed into several levels to remove more samples. First, the original signal *S*[*n*] is passed through a high-pass filter *H*[*n*] (equation (2)) and then the low-pass filter *L*[*n*] (equation (3)) is applied and can be shown as follows:

(2) $$\begin{array}{c} Y_{\text{high}}\left[k\right]=\sum_{n}S\left[n\right]\cdot H\left[2k-n\right], \end{array}$$

(3) $$\begin{array}{c} Y_{\text{low}}\left[k\right]=\sum_{n}S\left[n\right]\cdot L\left[2k-n\right], \end{array}$$

where *Y*_High_ and *Y*_low_ are the output of the algorithm after subsampling with factor 2, respectively. This operation is repeated at the next levels of decomposition.

Figure 4 shows the feature extraction operation where the main characteristics of the heartbeat are kept with 25 samples. After segmentation, the beat has decomposed into 4 levels using the DWT algorithm, and the number of signal samples has reduced at each level of decomposition. Finally, after the fourth level of decomposition, the number of heartbeat samples has reduced to 25 samples without losing the main beat information.

### 2.7. Classification

Classification is a two-step process. The first step is learning, in which a classifier is trained using training tuples on how to describe a set of class labels. The second step is to evaluate the classification model made in the previous step and use it for classification [43]. In this study, the training tuples involved in the building model are a set of features extracted from the signal in the data preprocessing stage, and class labels include normal heartbeat labels and atrial and RBBB arrhythmia labels.  Table 2 shows the number of tuples in the training dataset for each class label to create a classification model and the corresponding record in the MIT/BIH database. Since the number of class labels in this study is more than 2, we need to develop a multiclass classification model.

In machine learning, multiclass classification is a common problem in supervised learning. Multiclass classification is learned from a data set with *M* sample and *L* class label; each sample contains information in the form of the N attribute and the L?3. In this research, *M* = 5559, *N* = 25, and *L* = 3 are the parameters of classification models. Besides, several multiclass classifiers including decision tree, regression, and random forest have been trained due to their advantages and low computational complexity. Random Forest is an ensemble majority-vote-based classifier that uses a set of decision trees to classify data samples [44]. The set of decision trees forms a forest. During the classification, each tree decides its vote to identify the class, and finally, the most popular class with the most votes is selected for the current sample [44]. By evaluating the classification measures, the random forest model with 10 trees showed better performance than the other models and was selected as the final model. The multiclass random forest model was developed using the Apache Spark platform and was evaluated with a test dataset by the Spark Structured Streaming engine.

There are many reasons to choose a random forest model for classification, including its ensemble nature. Ensemble models are usually more accurate than nonensemble models. Also, the random forest model can be effectively applied to large datasets. Another feature of the random forest model is its ability to be used for future use and other data classifications. Finally, according to the specifications of ECG data in this study, the random forest classification model with its stated advantages could be one of the efficient models to achieve the desired goals in this research.

### 2.8. Online Classification Using Apache Spark

We have developed an online pipeline consisting of all of the aforementioned preprocessing and classification steps using existing functions at Apache Spark libraries and using the Spark structured stream processing engine to classification ECG streaming data and real-time cardiac arrhythmia detection.

### 2.9. Spark Structured Streaming

Structured Streaming is a powerful stream processing engine in Spark that is based on the Spark SQL engine [32]. Conceptually, Structured Streaming is capable of storing input streaming data with data frame API. The Structured Streaming considered sequential input data as an unlimited table, so it can benefit from the capabilities of Spark SQL in working with relational data, and our results are equivalent to performing a batch process across all input streaming data. Also, considering all input data as an unlimited table enables the user to run common data mining algorithms on streaming data [45].  Figure 5 shows the data stream schema in Structured Streaming top on the Apache Spark platform.

#### 2.9.1. File Source

There are several input sources for data entry in Structured Streaming, including the Kafka source and the file source. We used a file source to store the ECG test data as the input source. The data in the file source is entered with a time interval of 5 seconds, and by performing the calculations, the result of detecting the received beats in 5 seconds is generated from the received ECG record.

#### 2.9.2. Continuous Query

In an online environment, changes always happen suddenly. Therefore, it is not possible to react to changes with a traditional system and batch processing. In a streaming system, we can react timely to changes through a continuous query. This query is executed sequentially on the streaming data. The query execution time is defined by a predetermined time interval as the data is received [46]. The continuous query that we have implemented includes predefined pipeline steps that form the preprocessing and classification stages. In this study, the execution time of the query is considered based on a 5-second time interval, which means that every 5 seconds the query is executed once on the input streaming data.

#### 2.9.3. Real-Time Processing

The main steps in the real-time data processing of this research include the three steps of reading the data from the file source, running the pipeline and producing the results, and sending them to the database.

We have implemented our real-time computations using Structured Streaming through a continuous query with 5-second time intervals. Before starting to perform computations, the predeveloped random forest model is loaded for classification. After that, in the first stage of the computations, whenever the time interval is completed, 5 seconds of test data available in the file source are entered into the system through a continuous query; then in the second stage, the query commands are executed. And the predefined steps of data processing and classification are applied to the input data, respectively. Finally, in the third step, the results of the classification, which is the detection of arrhythmia class labels, are sent to the database. At subsequent time intervals, all of these steps are executed again on the input data, respectively, and continue until the data available in the file source are terminated.  Figure 6 shows the online pipeline proposed for cardiac arrhythmia detection using a machine learning model within the spark structured streaming framework.

### 2.10. Analysis Environment

We had a lot of hardware limitations to implement the steps of this research. To address these limitations, we launched our implementation tools in the Google Colaboratory environment on Google's virtual machine with a CPU of 2.3 GHz (single-core and two-threads), 12.6 gigabytes of RAM, and 100 gigabytes of disk space. In addition, our implementation stages are written in *Python* programming language version 3.6 and run on the Apache Spark platform version 2.4.3.

## 3. Results

### 3.1. Classification Statistics

Since the number of the class label in this study is more than 2 class labels, we have used multiclass classification evaluation metrics to validate our models. Sensitivity and specificity performance metrics were applied to validate the approach developed using test streaming data because of their compatibility with the nature of clinical data [22].

(4) $$\begin{array}{c} \text{sensitivity}:\frac{\text{TP}}{\text{TP}+\text{FN}}\times 100, \end{array}$$

(5) $$\begin{array}{c} \text{specificity}:\frac{\text{TN}}{\text{TN}+\text{FP}}\times 100. \end{array}$$

Table 3 shows the number of beats considered for test data sampled at 360 Hz for each class label, along with the corresponding record in the MIT/BIH database.

To validate our online arrhythmia detection approach, we used a 5-second packet of test streaming data for all records. Each cycle a 5-second time interval is completed, computations are performed on the received ECG data in this interval and the diagnostic results are recorded in the database.

We developed a decision tree, logistics regression, and random forest classification models using training data with 25 features (generated in the feature extraction phase). After validating these models with the test dataset, the random forest classifier based on an ensemble of 10 trees showed the best classification performance results. The overall results of multiclass classification metrics derived with this model are reported in Table 4.

Table 5 compares the classification performance of the proposed method with several approaches in the literature. It should be noted that the proposed approach is only compared with online approaches to arrhythmia diagnosis and offline approaches are not considered.

AUC stands for “Area under the ROC curve”. A ROC curve (receiver operating characteristic curve) is a plot showing the performance of a classification model at all classification thresholds. This curve plots two parameters: True Positive Rate and False Positive Rate. The higher the AUC value means that the model performs better in distinguishing between positive and negative classes. Therefore, if the AUC is equal to one, the model can perfectly distinguish between positive and negative classes. In this study, the AUC for the implemented multiclass model is 0.86 and shows that the model can distinguish three defined arrhythmia classes from each other with high performance.

In some of the methods listed in Table 5, only AF or RBBB or both arrhythmias are considered along with other arrhythmias. Also, other methods have used only two arrhythmia and nonarrhythmia class labels for diagnosis. Other online approaches [27, 29] have used AAMI annotations to detect what has not been considered in the comparison. Besides, the approach in [51] has used the Spark platform and focuses on data volume to offline cardiac arrhythmia detection which is not comparable to the results of this study. Also, in recent years, online and offline arrhythmia detection methods based on new approaches such as deep artificial neural networks have been introduced.  Table 6 shows the comparison of the performance metrics of our proposed method with the performance results of these methods.

### 3.2. Execution Time

In spark structured streaming it is possible to manage the query and prepare a report of all its specifications by the progress reporter, including the time spent by continuous queries from creation to completion. This time includes receiving the current batch offset, receiving the batch from the input source, query planning, and sending the batch result to the output at each round of query execution. Query planning time is the time required to implement pipeline, preprocessing, and classification steps. In this study, the time consumed to perform the query includes the time required to receive a 5-second batch of ECG data samples from the input source, the data preprocessing and the classification of the beats produced in this batch, and finally, the time is taken to send the detected class labels to the output sink.  Figure 7 shows the time spent in query consecutive execution on200 ECG packs. Accordingly, Table 7 compares the pipeline consumption time implemented in this study with the latest approaches presented by the researchers in real-time AF arrhythmia detection with an online approach. The pipeline developed in our proposed method is based on short 5-second epochs of ECG samples and a sampling rate of 360 Hz, but the approach presented in Sutton et al., 2018 is based on 1-minute epochs at 8 Hz sample rate. So to compare the total execution time of all the steps (reading data from a file source, preprocessing, classification) we set our pipeline based on 1-minute epochs time. So in this comparison, the number of our epochs has been reduced to 17 epochs at a 360 Hz sample rate.

According to the authors in Sutton et al., 2018, the high consumption time in this study is due to the time required to run the feature extraction algorithm in the preprocessing stage.

## 4. Discussion

Real-time data analysis techniques are divided into two general categories: algorithm-based and tool-based techniques. Most previous studies in this field are based on the use of algorithm-based techniques such as [19] for real-time *R* peak detection along with various machine learning algorithms for data classification. The most important algorithms used in these studies include decision tree, SVM, KNN, and neural networks classification algorithms. In this research, a tool-based technique based on a big data platform has been used for real-time analysis of ECG streaming data and implementation of traditional data classification algorithms. We use Apache Spark big data platform and Structured Streaming module, which, in addition to reducing computational delays, can keep the data stream as a relational table and supports SQL commands.

Compared to past research studies, this is the first study to use the Apache Spark Structured Streaming module for real-time cardiac signal analysis, which uses parallel processing to parallelize tasks in the diagnosis of heart disease.

In the past, many methods have been proposed for online ECG signal analysis and cardiac arrhythmia detection. In general, these methods are divided into two groups: algorithm-based and tool-based methods. Algorithm-based methods adopt a solution for dealing with timely analysis of streaming data. But in tool-based methods, it is the tool that enables real-time data stream analysis. Most of the methods developed in the past for online ECG signal analysis are traditional algorithm-based methods. However, these methods face many limitations. First, they need an expert to determine the heartbeat type and separate different beats [52]. Therefore, at this stage, the expert may make a mistake in diagnosing the heartbeat. Second, previous methods use techniques to extract the ECG signal features that are not able to extract all signal properties [52]. Thus, some important properties may be lost. All these limitations reduce the accuracy of the classification model [52].

With the development of machine learning algorithms, deep learning methods are widely used in cardiac arrhythmias detection [35–39]. Although deep learning methods can solve the limitations of traditional algorithm-based techniques in some areas such as learning important features, they also suffer from high computational complexity due to the lack of powerful hardware for model training [52]. Therefore, it is more reasonable to use deep learning methods in batch and offline processing to diagnose cardiac arrhythmias.

We used a technique based on the big data tool for significantly reducing the latency of the results. By defining user-defined functions, we have been able to run traditional algorithms that do not have high computational complexity on a big data platform. This capability avoids the computational complexity of deep learning methods and it maintains the classification performance metrics of previous models as the computational speed increases. Therefore, we have considered the advantages of the traditional algorithms and the state-of-the-art methods. It reduces the delay of the results as much as possible in addition to maintaining the classification measures. Our results show that the proposed method detects three types of cardiac arrhythmias with Average Consumption Time in about 1 second for all 5-second ECG signal epochs and 88.6% of accuracy, 83.8% of sensitivity, 86.01 of *F*1-score, 92.5% of precision, 97.5% of specification, and 86.23% of the total average of ROC score classification metrics.

Compared to online and offline methods presented in the past, our approach in addition to having the advantages of scalability, pipeline portability, and compatibility with other biological signals can significantly reduce latency in arrhythmia detection and maintain classification measures for precision, *F*1-score, specification, and AUC score.

On the other hand, compared to the tool-based methods [22], our results show better performance in terms of both classification performance and the amount of delay in producing results. This is due to the high-level API (Data Frame) provided by the Structured Streaming platform, which enables the implementation of fast SQL functions on streaming data. Also, Structured Streaming provides the user with a variety of output modes for generating results and output sinks to display it to minimize I/O operation latency.

In this study, three different classification algorithms, decision tree, random forest, and logistics regression, have been used, which can classify multiclass data. Each of the models developed in this study has other advantages in addition to the ability to classify multiclass data. The random forest model is usually more accurate than the nonensemble model because it is an ensemble and uses a combination of decision trees. Besides, the random forest model has a high ability to manage data with a large number of independent variables. However, in this study, the number of independent variables of each sample is relatively high and is 25 variables. Another advantage of a random forest classifier is that it can be stored for future use for other data classifications. Finally, according to the characteristics of ECG data in this study and their implementation environment for classification, a random forest model with its stated advantages could well be the most efficient model to achieve the desired goals in this research.

In recent years, the use of deep artificial neural network techniques in the volume [53–55] and high variety [56] of big data is increasing due to the need for large volumes of data to train models and its applications in data analysis with a complex structure [24]. However, the application of these methods in real-time data stream analysis with high production rates is less possible due to their high computational complexity [24]. A solution is an artificial neural network with incremental architecture [57, 58] in which the network structure changes with the arrival of new data. A new neuron is assigned to the network when a new sample arrives, and the network is being updated with new data. This method also faces the challenge of overadjusting network parameters and changing data distribution over time [24].

The loss of important ECG signal features in online cardiac arrhythmia detection methods can be partially addressed using deep learning approaches. Therefore, most of the methods proposed with deep artificial neural networks have been able to improve the classification performance metrics [35–39].

On the other hand, by implementing deep learning approaches on big data platforms and parallelizing computing, their computational complexity can be greatly reduced. Thus, an efficient method for real-time cardiac signal analysis to detect various arrhythmias is the integration of deep artificial neural network algorithms with important big data features (volume, variety, and velocity) that can overcome the limitations of existence online and offline ECG signal analysis techniques.

Unfortunately, none of the previous approaches specifically mention the rate of delay in diagnosing heart disease, and some of these other approaches that calculate the rate of delay do not have the same hardware as the hardware used in this study, so the results of these approaches in terms of delay the diagnosis of heart disease are not comparable to the delay in this study. However, the approach implemented in the earlier study, Sutton et al., 2018 [22], is one of the recent research studies and is very similar to our proposed approach due to the implementation of the random forest classifier Apache Spark Streaming (Not Structured Streaming) processing engine to diagnose AF arrhythmia. Therefore, it can be compared with our research in terms of time spent in diagnosing cardiac arrhythmias.

According to the results presented in Sutton et al., 2018 [22], which used a spark cluster with several nodes to implement the algorithms, the total amount of time consumed to execute all the implemented steps (calculation of PSPR features, calculation of descriptive features, and class prediction) of the research is close to two seconds, which is more than the time consumed to perform our research steps (Figure 7).

## 5. Conclusion

Our main goal in this study is to reduce the delay in real-time cardiac arrhythmias detection. We used the Structured Streaming stream processing engine to implement research steps with algorithms that do not have high computational complexity. Our results show a significant improvement in reducing latency and speeding up computing using the big data platform. In addition, our proposed approach is able to maintain the classification metrics compared to previous methods, despite the increase in the speed of computations.

### 5.1. The Major Contributions of This Research

Our proposed method is a tool-based method and provides capabilities that other algorithm-based methods do not have. These benefits include the following:

1. It reduces the delay in the real-time diagnosis of cardiac arrhythmias using parallel computing mechanism provided by the big data platform and the relative maintenance (or improvement) of multiclass classification performance compared to existing algorithm-based (or tool-based) methods (Tables 5–7)
2. Our online pipeline has the ability to real-time analyze other biological signals such as EEG signals
3. Our proposed method can adapt and integrate with different signal processing algorithms due to the implementation of user-defined functions
4. Our online pipeline is portable
5. Our online pipeline can be joined to static data (patient clinical symptoms) to increase the reliability of the results
6. Our streaming system is scalable and can accept new horizontal and vertical workers
7. Our streaming system is fault-tolerant with the concept exactly-once delivery and ensures that data is not lost if the system crashes, and by rebooting the system, results are generated immediately after the failure point

### 5.2. Significance Statement

We supply a novel machine learning pipeline for the real-time classification of AF and RBBB arrhythmias in - second ECG data intervals using a parallelized Apache Spark Structured Streaming Processing Engine.

We used the Pandas-UDF technique to implement classification and preprocessing algorithms on the new Apache Spark platform to implement preprocessing and real-time pipeline construction.

However, our proposed method faces limitations that could be key to further research in the future.

1. Our focus in this study is on the high-velocity feature of big data. If the variety feature is added to the data, the reliability of the results will increase for patients
2. This study aimed to reduce the final delay in the real-time diagnosis of cardiac arrhythmias. Therefore, in this research, the novel methods such as deep neural networks have not been used due to their high computational complexity
3. Our method still could not counter the concept drift in the real world. The concept drift refers to a change like data due to conditions such as noise. This phenomenon affects new features in online learning and can affect the accuracy of the results. Therefore, in the real world, it is necessary to provide a solution to deal with concept drift

### 5.3. Future Works

More studies can be done in the continuation of this research to be used with more confidence in the real environment and monitoring of heart patients.

An important event that may occur in streaming data is the concept of drift. This event refers to the change in the nature of the data over time, which may be based on noise or various environmental conditions. Using a mechanism to detect and deal with the drift while analyzing the signal could be a suggestion for the future. Another feature of big data is the high variety of data typing. This feature can be achieved by combining the patient's physiological characteristics along with the heart signals that are produced at high speed and indefinitely. These characteristics can include the patient's weight, sex, blood sugar, blood pressure, cholesterol levels, and other physiological characteristics of the patient. This can produce results with higher reliability that is closer to reality. Furthermore, the approach used in this research can be generalized to other streaming data. For example, it could be useful to use this approach to real-time analyze other signals produced in the body, such as the brain signal (Electroencephalography).

## Figures and Tables

**Figure 1:** Block diagram of data preprocessing and classification.

**Figure 2:** ECG filtered and R-peak detected of the signal in 360 Hz sample rate.

**Figure 3:** A normal segmented beat in 360 Hz sample rate.

**Figure 4:** Feature extraction of ECG signal using the DWT algorithm.

**Figure 5:** Data Stream as an unbounded table in Apache Spark Structured Streaming.

**Figure 6:** Framework of the proposed online cardiac arrhythmias detection pipeline on Apache Spark.

**Figure 7:** Execution time (Ms) consumed by a query for different packs in Apache Spark Structured Streaming.

**Table 1:** Record and number of the total samples considered for train and test datasets.

Data set	Record	Total samples
Train set	118-205-232	1111800
Test set	115-124-232	358200

**Table 2:** The number of training samples according to each class label sampled at 360 Hz and the corresponding record in the MIT/BIH database.

Class label	Record	Number of samples
Normal beat	205	400000
RBBB arrhythmia	118	400200
Atrial arrhythmia	232	311600

**Table 3:** The number of test samples according to each class label sampled at 360 Hz and the corresponding record in the MIT/BIH database.

Class label	Record	Number of samples
Normal beat	115	104400
RBBB arrhythmia	124	129600
Atrial arrhythmia	232	124200

**Table 4:** Multiclass classification metrics obtained using random forest on the test dataset.

Metrics	Accuracy (%)	Sensitivity (%)	Specificity (%)	F1-score (%)	Precision (%)	AUC score (%)	False positive rate
Value	88.7	83.8	97.5	86.08	92.5	86.2	0.024

**Table 5:** Classification performance of the proposed method and comparison with some online methods from the literature.

Method	Acc (%)	Se (%)	Sp (%)
Lee et al. [6]	99	—	—
Park and Kang [21]	96.7	99.5	89.9
Sutton et al. [22]	82.1	100	73.6
Lahdenoja [28]	97	93	100
Tateno and Glass [29]	—	94.4	97.2
Dash et al. [31]	—	90.2	91.2
Jang et al. [33]	91.9	84.6	94.3
Gradl et al. [47]	—	89.5	80.6
Leutheuser [48]	91.6	90.9	92.3
Yen et al. [49]	98.3	—	—
Oresko et al. [50]	93.3	—	—
Proposed method	88.7	83.8	97.5

**Table 6:** Classification performance of the proposed method and comparison with some recently proposed methods.

Approach	Method	Acc	Se/Rec	Pre	F1 score	Sp
Offline	Wang et al. [36]	—	82.2	83.8	82.8	—
	Ghosh et al. [35]	99.4	98.7	—	—	100
	Mahmud et al. [38]	99.2	99.1	99.0	99.1	—
	He et al. [39]	95.1	87.2	82.4	84.0	—

Online	Kanadala et al. [37]	—	74.2	—	—	88.4
	Proposed method	88.7	83.8	92.5	86.0	97.5

**Table 7:** Consumption time of the proposed method and comparison with the novel methods from the literature.

Methods	Implementation	Class number	Average consumption time for all epochs (s)	The number of epochs' sample	Epochs time (s)
Sutton et al., 2018 [22]	Apache Spark Streaming	2	±2	480 (8 Hz sample rate)	60
Sutton et al., 2018 [22]	MatLab	2	>2	480 (8 Hz sample rate)	60
Proposed method	Apache Structured Streaming	3	±1	1800 (360 Hz sample rate)	5

## Data Availability

The data utilized for finding the outcomes of this research have been taken from PhysioNet, and the well-known MIT/BIH arrhythmia database is available at https://archive.physionet.org/physiobank/database/mitdb/.
